# Carboplatin activates the cGAS-STING pathway by upregulating the TREX-1 (three prime repair exonuclease 1) expression in human melanoma

**DOI:** 10.1080/21655979.2021.1972198

**Published:** 2021-09-14

**Authors:** Zhourui Ma, Qianwei Xiong, Hongliang Xia, Wei Liu, Shu Dai, Shizhong Cai, Zhenhong Zhu, Xiangming Yan

**Affiliations:** a Department of Burns and Plastic Surgery, Children’s Hospital of Soochow University, Suzhou City, Jiangsu Province, China; b Department of Urology, Children’s Hospital of Soochow University, Suzhou City, Jiangsu Province, China; c Department of Child and Adolescent Healthcare, Children’s Hospital of Soochow University, Suzhou City, Jiangsu Province, China; d Department of Surgery, Children’s Hospital of Soochow University, Suzhou City, Jiangsu Province, China

**Keywords:** Apoptosis, carboplatin, metastatic melanoma, stimulator of interferon genes (STING), three-prime repair exonuclease 1 (TREX1)

## Abstract

Human melanoma is a highly aggressive type of cancer, causing significant mortalities despite the advances in treatment. Carboplatin is a cisplatin analog necessary for the treatment of various cancers and can also be used to treat human melanoma. We assessed the effects and mechanisms leading to inhibited proliferation and induced apoptosis of human melanoma after carboplatin therapy in vitro and in vivo. TREX1, cGAS/STING, and apoptotic protein expressions were determined through RT-qPCR and western blot assays. Cell proliferation was validated through MTT assays. The study used SK-MEL-1 and SK-HEP-1 tumor cell line inoculations along with carboplatin in nude mice to validate the results. The TREX1 levels were down-regulated in human melanoma cell lines. TREX1 overexpression-induced apoptosis and decreased proliferation in the human melanoma cell lines. TREX1 overexpression also activated the cGAS/STING pathway to induce apoptosis and decrease cell growth. Carboplatin activated TREX1, induced apoptosis, and decreased proliferation in the human melanoma cancerous cell lines. Finally, carboplatin reduced the in-vivo tumor size and weight. In conclusion, the study revealed that carboplatin activated TREX1 and cGAS/STING pathways to upregulate apoptosis. The work also provides in vitro and in vivo evidence to understand the effects of TREX overexpression on tumor suppression. Targeting of TREX1/cGAS/STING pathway could be an effective therapeutic alternative to human melanoma.

## 1. Introduction

Human Melanoma is a significantly aggressive tumor, responsible for at least 75% of skin cancer mortalities and increasing annual incidence [1]. The primary melanoma arises from malignant melanocyte transformation [2]. Primary tumor cells may metastasize through the lymphatic vessels, resulting in nodal tumor metastases, spreading further into the entire vascular system. The consequence of its continuous metastasis is the colonization of distant organs, such as lungs and brain [3]. Current melanoma therapies that focus mainly on the BRAF-targeted therapy (which involves down-regulating proteins of altered signaling pathways that occur in the affected individuals’ subset) often lead to resistance to treatment [4]. Despite the recent treatment progress through checkpoint inhibitors [5], approximately 70% of the patients with metastatic melanoma still do not respond to immunotherapies [6]. Consequently, a clear understanding of the cellular mechanisms that drive melanoma progression is needed to develop better therapeutic alternatives.

Cytosolic DNA sensing cGAS-STING (cyclic GMP-AMP synthase – stimulator of interferon genes) pathway is emerging as an essential mechanism that drives tumor growth driven by inflammation [7]. cGAS-STING chronic activation and its downstream effectors, for instance, TBK1, have been associated with inflammation persistence and cancer progression [8].

cGAS is a cytosolic sensor of DNA that initiates an immune response against microbial pathogens’ invasion, such as viruses [9]. In turn, cGAS activation induces the adapter protein STING, triggering interferon signaling [10]. The cGAS and STING homolog’s existence in eukaryotes and prokaryotes indicate an evolutionarily conserved mechanism of DNA sensing against pathogenic diseases [11]. Besides the cGAS and STING antimicrobial role, recent reports have expanded their functions to cancer, including other cellular roles like repair of DNA and autophagy [12].

The three-prime repair Exonuclease 1 (TREX1) is a 3ʹ⸻ 5ʹ DEDD family member, essential for replicating and repairing DNA. The TREX1 mutations have been associated with various complications, including systemic lupus erythematosus and cardiomyopathy [13]. Furthermore, TREX1 has been shown to prevent autoimmunity initiation through cytoplasmic ssDNA degradation [14]. The association between TREX1 and cancer has been reported, with research concluding that TREX1 targeting is a possible novel approach for cancer therapy. TREX1 is initiated by genotoxic stress and plays a critical role in melanoma and glioma cells’ protection to cancer drug therapies [15].

Carboplatin (1, 1-cyclobutanedicarboxylic acid (C_6_H_12_N_2_O_4_Pt) is a second-generation platinum anti-tumor drug derived from cisplatin. The compound forms an intra-stand and inter-strand cross-linking with a cell, leading to the modification of DNA structure and DNA synthesis arrest. Carboplatin has been used singly or in combination with various agents, such as Bortezomib or Paclitaxel to treat malignant melanoma or small lung cancers [16,17]. Furthermore, carboplatin has been reported as a suitable neoadjuvant chemotherapy in Triple negative Breast Cancer (TNBC) [18]. However, no studies have assessed the role of carboplatin as a STING agonist and further investigations are required to provide a complete understanding of the role of carboplatin in melanoma suppression, and the activation of TREX-1 and cGAS/STING pathways. The present investigation hypothesized that carboplatin activates the cGAS-STING pathway through the upregulation of the TREX-1 expression in human melanoma. This study aimed at assessing the expression of TREX1 in human melanoma and the effects of its overexpression on the cGAS-STING pathway and human melanoma proliferation. Finally, the role of carboplatin on human melanoma proliferation in vitro and in vivo was determined.

## 2. Materials and methods

### 2.1. Human specimens

The research strictly followed the Helsinki Declaration. Our school’s local committee for ethics permitted the research. All participants in this study have given written informed consent. For tumor specimen collection, a biopsy was performed to collect human sinonasal mucosal melanoma (10 specimens) and adjacent tissue as control. Pre-informed permission was received before the biopsy. Samples were stored at a − 80°C refrigerator.

### 2.2. Cell culture

Tumor SK-HEP-1, SK-MEL-1, A375, MV3, and the control HPM cell line were obtained from the Chinese Academy of Science Biobank and cultured in DMEM supplemented with 10% FBS and Penicillin-streptomycin. The condition of cell culture was 37°C and 5% CO_2._ Change of media was done after every 48 hours.

### 2.3. Transfection

SK-MEL-1 and SK-HEP-1 cells experimental cells were divided into two groups, each then transfected using TREX1-OE and the comparable controls (pcDNA), respectively. The plasmids were synthesized from Genepharma (Shanghai). Each group contained approximately 3 × 10^5^ cells. Transient transfection of cells was done using Lipofectamine 2000^TM^ (Invitrogen, Carlsbad, CA, USA). In brief, when the cells were at a confluence of 70%, they were plated in 6-well plates and transfected using the appropriate plasmids.

### 2.4. RNA isolation

Total RNA was extracted from SK-HEP-1 and SK-MEL-1 cells treated with Carboplatin or 0.1% DMSO (vehicle) for 24 h using Trizol Reagent (Invitrogen, CA, USA) as per the manufacturer’s instructions. Samples of RNA were carefully dissolved through an incubation for 10 min at 55°C. Contamination of DNA was eliminated by the DNase I (Invitrogen) treatment at 37°C for 30 min, followed by the DNase I heat inactivation before being quantified using a Nano-Drop spectrophotometer. The storage condition of purified RNA was at −80°C for further use.

### 2.5. Synthesis of cDNA and real-time qRT-PCR

The first-strand cDNA synthesis was done with the iScriptTM cDNA synthesis kit (Biorad) per the manufacturer’s instructions. The obtained cDNA was used to carry out RT-qPCR (Bio-Rad iCycler iQ5TM Real-Time PCR detection system) using 2X iQ SYBR Supermix (Invitrogen). The primer sequences (from 5ʹ end to 3ʹ end) used for qRT-PCR are as follows:

TREX1-F-GAGAGTGTGCAGCCGAGTCA, R-AGATGAGGGTCTGCATGGGC.

Β-Actin-F-GTGGGCA TGGGTCAGAAG, β-Actin-R-TCCATCACGATGCCAGTG.

The levels of gene expression were assessed by the cycle threshold (Ct) method. Mean values of Ct from duplicate results were used to calculate the target gene expression with housekeeping gene normalization. The difference in the fold expression was finally calculated through the ΔΔC_t_ method.

### 2.6. Cell viability

Cell proliferation assay was conducted using 3-(4, 5-Dimethylthiazol-2-)-2,5-diphenyl tetrazolium bromide (MTT) [19]. About 1 × 10^4^ cells/well were plated in 96-well plates and cultured at 37°C for numerous time intervals. After washing the cells, 20 µl MTT reagent was added per well. The cells were further grown for 4 h. Afterward, DMSO (150 µl) was added after the removal of MTT. Finally, the optical cell density (OD) was determined in a microplate reader at 562 nm.

### 2.7. Determination of apoptosis

To detect carboplatin-induced apoptosis, annexed V/PI double staining combined with flow cytometry was used. Exponentially proliferating SK-MEL-1 or SK-HEP-1 cells were treated with 80 µM of Carboplatin and analyzed 72 h later. The tumor cells were trypsinized and combined with the free-floating cells in the supernatant. Later, the cells were washed in cold PBS and stained with annexin V FITC following the manufacturer’s guidelines (BD PharMingen). The fraction of Sub-G1 was determined through flow cytometry [15]. The assays were repeated at least three times. The mean values ± SD were determined, and a statistical data analysis was done using Student’s t-test.

### 2.8. Western blot analysis

Extraction of proteins from tumor cells was done using RIPA lysis buffer (Beyotime, Shanghai, China). The concentration of protein was assessed using a BCA protein kit (Beyotime). Separation of aliquots of protein was then done using SDS-PAGE (12%). The separated proteins were later transferred to polyvinylidene fluoride (PVDF) membranes (Millipore, Billerica, MA, USA) and blocked using PBS containing 5% milk and 0.1% Triton X-100. After blocking, the membrane was then incubated with anti-Trex1, -cGAS, -STING – cytochrome C, – BAX, -Tubulin, -TBK1, -p-TBK1, -IRF3, -p-IRF3, -p65, -AKT, -p-Akt, and -DasbA-L primary antibodies (1:1,000) overnight at 4°C. Antibodies against GAPDH were used as the internal control. The incubation of the membrane with appropriate HRP-conjugated secondary antibodies (1:10,000) was then done. Finally, the bands were pictured using Immobilon^TM^ HRP substrate (Millipore).

### 2.9. In vivo *experimental mouse model*

The 32 Balb/c mice (male, 8 weeks-old, and 20 g in weight) were acquired from the Children’s Hospital of Soochow University. The animal experiment research protocol was approved by the Ethics Committee of Children’s hospital of Soochow University and performed under the ‘Guidelines for the care and use of experimental animals.’

SK-MEL-1 or SK-HEP-1 cells in the log phase were harvested and then suspended in cold PBS to a concentration of 2.5 × 10^6^ cells/mL. Later, 100 µl of the cell suspension was injected into all experimental animals’ right posterior flank (16 mice for each cell line) to obtain a solid tumor growth. Five days after inoculation with each tumor cell, the mice were randomly assigned to two groups, each with eight animals (for each cell line). The animals were intraperitoneally injected with the drug for three cycles after every 7 days. Each treatment group received Carboplatin (100 mg/kg), while the control group was administered with saline (100 µL of saline 0.9%). The dosage of Carboplatin was based on Souza et al. [20]. The tumor size and body weight were periodically determined.

Tumor measurements were determined by a caliper ruler. The tumor volume was determined by the equation: tumor volume (mm^3^) = (length × width^2^)/2. The length and the width were presented in millimeters [21]. The necropsy was done after 26 days by removal of tumors that were removed with the removal of the tumor.

### 2.10. Statistical analysis

The mRNA profile of TREX1 and its corresponding survival data were retrieved and analyzed from The Cancer Genome Atlas (TCGA) database available at cbioportal (https://www.cbioportal.org/).

### 2.11. Statistical analysis

Data analysis was done using Graph Pad prism. The results are presented as the mean ± SD from three independent results. P values ≤0.05 derived by student’s t-test were considered significant.

## 3. Results

### 3.1. TREX1 is downregulated in the human melanoma cancer

Human melanoma is a highly aggressive type of cancer, causing significant mortalities despite the advances in treatment. Carboplatin is a cisplatin analog used for the treatment of various cancers. The current investigation postulated that carboplatin can suppress human melanoma through the activation of the cGAS-STING pathway via TREX-1 upregulation. First, we used TCGA database to evaluate the role of TREX1 in human melanoma. The results showed that TREX1 expression was associated with poor prognosis and low survival rate. Further, western blot and RT-qPCR experiments were used to determine the expression of TREX1 and mRNA in A375, SK-HEP-1, SK-MEL-1, and MV3 tumor and the HPM normal cells. According to the western blot and RT-qPCR findings, the expression of TREX1 is higher in HPM cells, but significantly reduced in the A375, SK-HEP-1, SK-MEL-1, and MV3 tumor cell lines, as shown in Figure 1(a,b). In addition, we determined the expression of TREX1 in human sinonasal mucosal melanoma tissues. Similarly, the observations indicated a significant reduction in TREX1 expression in tumor tissues compared to the control tissues, as shown in Figure 1(c). Determination of mRNA expression in tumor tissues through RT-qPCR also confirmed significant downregulation of TREX1 mRNA in tumor tissues compared to the adjacent control tissues (Figure 1(d)).

**Figure 1.** TREX1 is downregulated in the human melanoma cancer

(a): Survival plot of TREX1 expression level and alteration in melanoma patient survival. (b): Western blot analysis representing expression of TREX1 in human melanoma cancer cell lines. (c): RT-qPCR analysis representing expression of TREX1 in human melanoma cancer cell lines. (d): Western blot analysis representing expression of TREX1 in human melanoma clinical specimens. (e): RT-qPCR analysis representing expression of TREX1 in human melanoma clinical specimens. (* = p > 0.05)

### 3.2. Overexpression of TREX-1 induce apoptosis and decrease proliferation in human melanoma, cancerous cell lines

To determine the effects of TREX1 overexpression in human melanoma, SK-HEP-1 and SK-MEL-1 cancerous cell lines were transfected with TREX1 overexpression plasmids, and the effects of overexpression were assessed through western blot and RT-qPCR. Our observations indicated an increased TREX1 protein and mRNA expression in SK-MEL-1 cells in a time-dependent manner, with the highest expression observed after 48 h (Figure 2(a,Figure 2b)). Similarly, the TREX1 protein and mRNA levels were significantly increased in SK-HEP-1 cells in a similar pattern (Figure 2(c,Figure 2d)). To determine the effect of TREX1 overexpression on apoptosis, we used annexin V/PI double staining kit and flow cytometry analysis. We observed a significantly increased apoptotic cell following the overexpression of TREX1 in both the SK-MEL-1 and SK-HEP-1 cells (Figure 2(e,Figure 2g)). Cell proliferation experiments through MTT confirmed a significantly inhibited cell growth following the TREX1 overexpression in the SK-MEL-1 and SK-HEP-1 cells (Figure 2(f,Figure 2h)).

**Figure 2.** Overexpression of TREX1 induce apoptosis and decrease proliferation in human melanoma, cancerous cell lines

(a): Western blot analysis representing expression of TREX1 after transfection of TREX1 overexpression plasmid in SK-MEL-1 cell line. (b): RT-qPCR analysis representing expression of TREX1 after transfection of TREX1 overexpression plasmid in SK-MEL-1 cell line. (c): Western blot analysis representing expression of TREX1 after transfection of TREX1 overexpression plasmid in SK-HEP-1 cell line. (d): RT-qPCR analysis representing expression of TREX1 after transfection of TREX1 overexpression plasmid in SK-HEP-1 cell line. (e): Flow cytometry analysis representing the apoptosis rate after transfection of TREX1 overexpression plasmid in SK-MEL-1 cell line. (f): MTT analysis representing cell viability rate after transfection of TREX1 overexpression plasmid in SK-MEL-1 cell line. (g): Flow cytometry analysis representing apoptosis rate after transfection of TREX1 overexpression plasmid in SK-HEP-1 cell line. (h): MTT analysis representing cell viability rate after transfection of TREX1 overexpression plasmid in SK-HEP-1 cell line. (* = p > 0.05)

### 3.3. Overexpression of TREX1 activates the cGAS/STING pathway to induce apoptosis and decrease cell growth

Next, we aimed to investigate the mechanism of apoptosis induction by TREX-1. We analyzed the expression of cGAs and STING expressions through western blotting and RT-qPCR. Our observations indicate an increased expression of both cGAs and STING in a time-dependent manner, with the highest expression observed after 48 h in both SK-MEL-1 and SK-HEP-1 cells (3A and 3B). Further investigations showed increased expressions of p-TBK1, p-p65, p65, TNFa, p-IRF3, DasbA-L, and Tubulin following the overexpression of TREX1 in SK-MEL-1 cells, as shown in Figure 3(c). The investigation of apoptosis through western blot also indicated increased Caspase 3, BAX, cytochrome C, and p-AKT following the TREX overexpression in SK-MEL-1 cells, as shown in Figure 3(d).

**Figure 3.** Overexpression of TREX1 activates the cGAS/STING pathway to induce apoptosis and decrease cell growth

(a): Western blot analysis representing expression of cGAS & STING after overexpression of TREX1 in SK-MEL-1 cell line. (b): Western blot analysis representing expression of cGAS & STING after overexpression of TREX1 in SK-HEP-1 cell line. (c): Western blot analysis representing involvement of TREX1 overexpression in regulating cGAS/STING pathway in SK-MEL-1 cell line. (d): Western blot analysis representing involvement of TREX1 overexpression in regulating pathways involved in apoptosis and cell growth in SK-MEL-1 cell line. (* = p > 0.05)

### 3.4. Carboplatin activates TREX1 and induce apoptosis and decrease proliferation in human melanoma, cancerous cell lines

To investigate the effects of carboplatin on apoptosis, the cancerous cell lines were treated with various doses of Carboplatin (10 µM, 20 µM, 40 µM, and 80 µM) for 72 h and the expressions of TREX were analyzed through western blotting and RT-qPCR. The observations indicated an upregulated expression of TREX1 in a carboplatin-dose-dependent manner, with the peak observed at 80 µM in SK-MEL-1 and SK-HEP-1 cells, Figure 4(a-b). Further, treatment with carboplatin induced a significant increase in the expressions of cGAS/STING/p-TBK1/TNFa/p-IRF3 and the apoptosis protein Caspase 3, Bax, caspase 3, and p-AKT, as shown in Figure 4(c,d), respectively. Apoptosis study through flow cytometry also showed a significant increase in apoptotic cell populations after treatment with carboplatin in both SK-HEP-1 and SK-MEL-1, as shown in Figure 4(e,Figure 4g), respectively. Carboplatin treatment also led to a significantly reduced proliferation of SK-HEP-1 and SK-MEL1 cells, as shown in Figure 4(f,Figure 4h), respectively.

**Figure 4.** Carboplatin activates TREX1 and induce apoptosis and decrease proliferation in human melanoma through cGAS/STING pathway

(a): Western blot analysis representing the expression of cGAS & STING after carboplatin stimulation in SK-MEL-1 cell line. (b): Western blot analysis representing the expressionof cGAS & STING after after carboplatin stimulation in SK-HEP-1 cell line. (c): Western blot analysis representing the involvement of carboplatin in regulating the cGAS/STING pathway in the SK-MEL-1 cell line. (d): Western blot analysis representing the involvement of carboplatin in regulating pathways involved in apoptosis and cell growth in the SK-MEL-1 cell line. (e): Flow cytometry analysis representing apoptosis rate after carboplatin stimulation in SK-MEL-1 cell line. (f): MTT analysis representing cell viability rate after carboplatin stimulation in SK-MEL-1 cell line. (g): Flow cytometry analysis representing apoptosis rate after carboplatin stimulation in SK-HEP-1 cell line. (h): MTT analysis representing cell viability rate after carboplatin stimulation in SK-HEP-1 cell line. (* = p > 0.05)

### 3.5. Carboplatin reduces the in-vivo tumor size and volume

Finally, we investigate the effects of carboplatin in human melanoma in vivo. Following the injections of Balb/c mice with tumor cells and subsequent treatments with 100 mg/kg carboplatin, the tumor appearance, volume, and weights were significantly reduced in the animals injected with SK-HEP-1 tumor cells (Figure 5a-Figure 5c). Similar observations were made following injections of mice with SK-MEL-1 cells and the subsequent carboplatin treatments, as shown in Figure 5(d-Figure 5f). Taken together, these data confirm the suppressive function of carboplatin in human melanoma proliferation through cGAS/STING pathway activation.

**Figure 5.** Carboplatin treatment reduces the in-vivo tumor size and volume

(a): Visual observation of tumor size in nude mice inoculated with SK-MEL-1 cell line along with carboplatin treatment. (b): Comparison of tumor volume (mm^3^) in nude mice inoculated with SK-MEL-1 cell line along with carboplatin treatment. (c): Comparison of tumor weight (g) in nude mice inoculated with SK-MEL-1 cell line along with carboplatin treatment. (d): Visual observation of tumor size in nude mice inoculated with SK-HEP-1 cell line along with carboplatin treatment. (e): Comparison of tumor volume (mm^3^) in nude mice inoculated with SK-HEP-1 cell line along with carboplatin treatment. (f): Comparison of tumor weight (g) in nude mice inoculated with SK-HEP-1 cell line along with carboplatin treatment. (* = p > 0.05)

## 4. Discussion

Human melanomas are examples of neoplasms with highly rising incidences. Compared to localized tumors, which are generally cured through surgery, metastatic melanomas present a poor prognosis and no durable response to conventional treatment [22]. In addition, chemotherapeutic approaches are linked to resistance to drugs and harmful side effects. As such, the development of more efficient and novel treatments for human melanoma is necessary. The current research investigated Carboplatin’s role in the treatment of human melanoma. This study further investigated the expression of TREX1 in human sinonasal mucosal melanoma (SNMM) tissues. SNMM is a rare cancer that comprise less than 10% of the sinonasal cancers. About 70% of SNMM are found in the nasal cavity, while 14% occur in the maxillary sinus, and typically occur as black patches [23]. SNMM generally harbors an extremely poor prognosis with a less than 30% 5-year survival. The SNMM subtype may be biologically different from the most common cutaneous one. The findings reported that carboplatin activates TREX1 and cGAS/STING, leading to the suppression of proliferation in human melanoma.

TREX1 activity is reduced in various cancers, for instance, pancreatic [24], gastric [25], and cervical cancer [26]. Additionally, reports have shown that treating cancerous cells in vitro using UV-light, or different genotoxic anti-tumor agents is linked to the elevation of TREX1, and TREX1 siRNA knockdown initiates tumor cell deaths post-treatment [15]. Similarly, our findings indicated reduced TREX1 expressions in human melanoma cancer as was expressed in A375, SK-HEP-1, SK-MEL-1, and MV3 tumor cell lines. Mutations in TREX1 have also been associated with other diseases, such as retinol vasculopathy with cerebral leukodystrophy (RVCL) and Familial Chilblain Lupus [27].

TREX1 overexpression affects the cGAS/STING pathway. TREX1 plays an upstream regulatory role in anti-tumor response mediated by radiation. The expression of TREX1 depends on the drug dosage treatment; hence, it is being overexpressed to suppress the tumor. TREX1 expression is initiated at a sufficient level for degrading DNA, which can accumulate in the cytosolic region of the treated tumor cell, precluding interferon (IFN-1) pathway activation induced through cyclic GMP-AMP (cGAMP) synthase (cGAs) and the associated downstream adaptor STING [28]. In agreement with these findings, following an overexpression of TREX1, our results indicated an increased expression of both cGAs and STING in a time-dependent manner, with the highest expression observed after 48 h in both SK-HEP1 and SK-MEL-1 cells. On activation, STING moves to the Golgi apparatus, recruiting Tank Binding Kinase 1 (TBK1), leading to its phosphorylation [29]. The Phosphorylated STING recruits the IRF3 to be phosphorylated by TBK1. Finally, activated IRF3 dimerizes then translocates to the nucleus, promoting the IFN expression [30]. Our results also confirmed the increased expressions of p-TBK1, p-p65, p65, TNFa, p-IRF3, DasbA-L, and Tubulin following TREX1 overexpression.

Carboplatin is a DNA damaging cisplatin agent [22] which induces TREX1 expression at a higher dosage, consequently inducing apoptosis. In agreement, our results demonstrate that treatment with carboplatin leads to increased expressions of cGAS/STING/p-TBK1/TNFa/p-IRF3 and the apoptosis protein Caspase 3, Bax, caspase 3, and p-AKT. Carboplatin treatment also initiated apoptosis in vivo by binding to the nuclear DNA, resulting in various structural adducts and activating various cellular responses, such as transcription inhibition [20]. In the in vivo experiments, Carboplatin’s anti-tumor response was confirmed by significantly inhibiting tumor appearance, volume, and weights.

Summarily, this study gives a noble view on the role of carboplatin in suppressing human melanoma. TREX1 is downregulated in human melanoma, overexpression of TREX1 induces apoptosis and decreases proliferation in human melanoma cancerous cell lines, TREX1 overexpression activates the cGAS/STING pathway to induce apoptosis and decrease cell growth. Carboplatin activates TREX1, induces apoptosis, and decreases proliferation in the human melanoma cancerous cell lines. Finally, this study shows that carboplatin reduces the in-vivo tumor size.

## 5. Conclusion

The work also provides in vitro and in vivo evidence to understand the effects of TREX on tumor suppression. Our study illustrated that the level of TREX1 is lowered in human melanoma. Moreover, an increase in TREX1 activates the cGAS/STING pathway to induce apoptosis and decrease cell growth. Finally, we conclude that carboplatin activates TREX1 and cGAS/STING pathways to upregulate apoptosis. Targeting of TREX1/cGAS/STING pathway using carboplatin could be a novel and an effective therapeutic alternative for human melanoma.

## Research highlights

- TREX1 overexpression activates the cGAS/STING pathway and induces human melanoma apoptosis.
- Carboplatin activates TREX1 and induces apoptosis and decreases proliferation in human melanoma and cancerous cell lines.
- Carboplatin suppresses tumor size and volume in vivo
